# Effects of Neurodynamic Mobilization on Health-Related Quality of Life and Cervical Deep Flexors Endurance in Patients of Cervical Radiculopathy: A Randomized Trial

**DOI:** 10.1155/2022/9385459

**Published:** 2022-10-05

**Authors:** Shazia Rafiq, Hamayun Zafar, Syed Amir Gillani, Muhammad Sharif Waqas, Sidrah Liaqat, Amna Zia, Yasir Rafiq

**Affiliations:** ^1^Physiotherapy department Jinnah Hospital, Lahore, Pakistan; ^2^Department of Odontology, Clinical Oral Physiology, Faculty of Medicine, Umea University, Umea, Sweden; ^3^University Institute of Physical Therapy, University of Lahore, Lahore, Pakistan; ^4^College of Applied Medical Sciences, Rehabilitation Research Chair, Department of Odontology, Clinical Oral Physiology, Faculty of Medicine, King Saud University, Riyadh, Saudi Arabia; ^5^Allied Health Science, University of Lahore, Lahore, Pakistan; ^6^Services Hospital, Lahore, Pakistan; ^7^Physiotherapy Department, Mayo Hospital, Lahore, Pakistan; ^8^Pathology Department, Combined Military Hospital, Kohat, Pakistan

## Abstract

**Purpose:**

Cervical radiculopathy is disorder of cervical spinal nerve root affecting large number of population. Previously many studies are conducted to design suitable protocol for management of this disorder, but they lack in quality. The purpose of this study was to compare the effects of neural mobilization and cervical isometrics on health-related quality of life and deep flexors endurance in cervical radiculopathy.

**Methods:**

A double-blinded randomized clinical trial was conducted at Mayo Hospital, Lahore, Pakistan. Eighty-eight patients within the age range of 35-50 years were included in the study after taking their consent. In the experimental group (*n* = 44), median nerve mobilization was applied along with cervical isometric exercises. The control group (*n* = 44) performed cervical isometric exercises alone. Muscle endurance was measured by craniocervical flexion test and quality of life on 36 items short form health survey SF-36 scale. Measurements were taken at baseline, at 2^nd^ week, and at 4^th^ week. For missing data, intention-to-treat analysis was used.

**Results:**

Within-group comparison with Friedman test showed a significant difference between pre, mid, and posttreatment scores on craniocervical flexion test and in all domains of SF 36 in both groups. While between-group comparison with Mann–Whitney *U* test showed all variables were similar at baseline but after 4 weeks there was a statistically significant improvement in craniocervical flexion test scores and all domains of SF 36 in the experimental group. But domain of pain showed mean rank of 49.43 after 4 weeks in the experimental group and 39.57 in the control group with *p* = 0.065 and *d* = 0.579, while for all the other 7 domains values were *p* < .05 and *d* > 0.25.

**Conclusion:**

Neural mobilization combined with cervical isometrics shows significant effects in improving quality of life and deep flexors endurance in patients with cervical radiculopathy than cervical isometrics alone.

## 1. Introduction

Cervical radiculopathy impacts cervical nerves roots, with the highest prevalence of C6 and C7 nerve roots. Inflammation or impingement of these nerve roots trigger pain receptors present in soft tissues and joints of the cervical spine, leading to sensory changes such as tingling and motor loss in dermatomal and myotomal distribution depending on affected nerve root. Patients often complain of neck pain but usually they seek treatment for radiating pain in the arm [1–3].

Factors that can cause cervical radiculopathy are overuse injuries of the neck, inappropriate posture during exercises, degenerative disc disease, osteophytes formation, and road-side accidents [4]. Especially in developing countries like Pakistan, people suffer from various physical, mental, and social issues. These factors result in feeble bones, frail muscles, weak immunity, and deteriorated body mechanics which leads to spinal and musculoskeletal problems [5].

For the diagnosis of cervical radiculopathy magnetic resonance imaging is used as gold standard. As this is not readily available in all the medical facilities so manual diagnostic tools like Spurling's test, upper limb neurodynamic test 1, distraction test, and ipsilateral cervical rotation test are used in this study. Criteria devised by Wainner et al. is used, which is based on four variables and have a specificity of 94% [6].

Despite lack of evidence about the best nonsurgical technique for treatment of cervical radiculopathy, there are methods shown to be effective in reducing pain and discomfort. Strengthening exercises, muscle energy techniques, manual techniques, and the use of electrophysical modalities like hot packs, ultrasound, infrareds, laser, cryotherapy, transcutaneous electrical nerve stimulation TENS have shown to be effective in improving range of motion, reducing pain, and increasing muscular strength [7]. Another technique that is used is neural mobilization, which is based on the concept of neuro-dynamics by Shacklock. This approach influences physiology of pain through mechanical treatment of neural tissues and the surrounding structures of nervous system. The main aim is to restore the disturbed dynamic balance between the neural tissues and surrounding nonneural tissues. This will permit decrease pressure on the neural tissues and enhance optimal physiological functioning [8, 9].

Literature shows that exercise intervention containing isometrics of cervical muscles alleviates pain and disability [10, 11]. Physical activity in the form of exercises has supporting evidence of improving sleep, emotional, physical, and cognitive functioning status by reducing depression and anxiety, this in turn impacts the quality of life positively [12, 13]. In the past, many studies have been conducted on the treatment of cervical radiculopathy but the majority of these show limitations in quality of the study, treatment methods, and inappropriate inclusion criteria [14]. This lack of evidence warrants further investigation.

Therefore, it is necessary to figure out the best way to manage cervical radiculopathy. This study is focused on aspects of cervical muscular endurance and quality of life of patients with cervical radiculopathy and evaluates the effectiveness of neurodynamic mobilization technique.

## 2. Method

### 2.1. Study Design

A parallel-group randomized trial according to consolidated standards of reporting trial (CONSORT) guidelines was conducted with intention-to-treat analysis as shown in Figure 1. Participants were included from Physiotherapy Department Mayo Hospital Lahore, Pakistan. After confirming the inclusion criteria, participants willing to participate were randomly allocated into two groups.

### 2.2. Sample Size

Sample was calculated using G∗Power software. 88patients (44 in Group A and 44 in Group B) were included in the study using effect size 0.70, calculated from previously reported difference in a study by Sambyal and Kumar [4] using mean ± SD, at level of significance 0.05 and power 90%.

### 2.3. Participants and Setting

Participants were included from Physiotherapy Department Mayo Hospital Lahore, Pakistan. Subjects were included if positive results were found in a minimum three of four tests (Spurling's test, Upper Limb Neurodynamic Test 1, Distraction test, and ipsilateral cervical rotation of less than 60^0^) [6].

Both male and female participants between the ages of 35-50 years, having radiating symptoms of cervical radiculopathy with no previous history of cervical surgeries, and no loss of upper limb movement were included in the study. Subjects having traumatic history, osteoporosis, hypermobility, cervical circulatory disorders, peripheral nerve entrapment, and malignancy were excluded from study.

### 2.4. Randomization and Blinding

In this randomized controlled trial simple random sampling technique was used with 1 : 1 allocation. Participants were randomly allocated into two groups by computerized generated randomization table. Concealment of allocation was achieved through sequentially numbered opaque sealed envelopes (SNOSE) method according to guidelines of Doig and Simpson [15]. Envelops were made by an independent researcher with no clinical involvement.

Patient, assessors, and data analysts were blinded to allocation of treatment groups in this study. Except for the therapist, all other staff was kept blinded as they were not informed about the details of allocation. Trial adhered to established procedures to maintain separation between staff who was collecting outcome measurements and the therapist. Patients were blinded to treatment allocation as treatment was given in separate rooms for each group. A therapist who is not blinded did not take the outcome measurements. All the other assessors, investigators, and analysts did not know the details of treatment.

### 2.5. Intervention

In the experimental group, the neural mobilization sliding technique was given for the median nerve along with cervical isometric exercises. Neural mobilization was done according to technique described by Butler [16]. The subject was placed in supine position and slider neural mobilization of the median nerve was given. The sequence of treatment for median nerve was glenohumeral abduction and external rotation, forearm supination, wrist extension, elbow extension, and neck side bending to opposite side. This sequence was repeated with a hold of three seconds with ten repetitions. Cervical isometric exercises were given with patient in sitting position. Three sets of these exercises were performed with ten repetitions in each direction with 5 second hold [4]. Hot pack was applied to all participants for ten minutes.

In the control group, only three sets of cervical isometric exercises were applied with ten repetitions in each direction with five second hold. Hot pack was given for ten minutes to all participants before treatment.

In both groups treatment duration lasted for 30 to 40 minutes per session. Participants were treated three times per week for four weeks. Measurements were taken at the baseline before starting treatment, then after two weeks, and finally after fourth week of treatment.

### 2.6. Outcome Measures

The outcomes were to measure the effectiveness of the neural mobilization technique on cervical muscle endurance and quality of life. Muscle endurance was measured by using the craniocervical flexion test (CCFT). CCFT was performed with the patient in crook lying position. An uninflated pressure sensor was placed behind the upper cervical spine and then inflated to baseline pressure of 20 mmHg. The patient was instructed to perform a nodding movement while examiner provided visual feedback. Measurements were taken to measure any change in the pressure gauge [17].

Quality of life was measured by 36 items short form health survey SF-36. That included physical functioning, bodily pain, role limitations due to physical health problems, role limitations due to personal or emotional problems, emotional well-being, social functioning, energy/fatigue, and general health perceptions. Few other variables of this research are also present in the preprints article at research square [18].

### 2.7. Statistical Analysis

Data were analyzed using Statistical Package for Social Sciences (SPSS) version 21 program. Descriptive analyses (mean and standard deviation) were performed for continuous variables. Frequencies and percentages were calculated for categorical variables. Data were analyzed for normality by applying the Shapiro-Wilk test. Friedman test was used for within-group analysis. For the post hoc test to determine where the differences actually occur, Wilcoxon signed-rank tests on the different combinations (premid, midpost, and prepost) of related groups were used. Mann–Whitney *U* test was used for between-group comparisons. Intention-to-treat analysis with the technique of last observation carried forward (LOCF) was used to handle the missing data due to loss of follow-up.

## 3. Results

### 3.1. The Flow of Participants, Therapists, and Centers Through the Study

Eighty-eight participants were recruited who underwent baseline testing. Randomization allocated forty-four participants to the experimental group (neural mobilization) and forty-four to the control group (conventional treatment). The mean age of the subject in the experimental group was 41.09 ± 6.05 and the control group was 42.22 ± 5.62. According to the gender distribution in the neural mobilization group, 15 (34.1%) were males and 29 (65.9%) were females and in the conventional treatment group, 13 (29.5%) were males and 31 (70.5%) were females.

Participants completed intervention as allocated and measurements were taken at baseline, after the second week then final postassessment at the fourth week.

There was the loss of follow-up of two participants from the experimental group and of three participants from the control group. Participants discontinued intervention due to an uncertain pandemic situation.

Sessions were provided by the physiotherapist who had twenty years of experience. Pre and post evaluations were done by physiotherapists who had at least five years of experience.

Only one center Department of Physiotherapy, Mayo Hospital Lahore, Pakistan was involved in the study.

### 3.2. Compliance with the Trial Method

There was loss of follow-up of two participants from the experimental group and of three participants from the control group. Participants discontinued intervention due to an uncertain pandemic situation.

### 3.3. Effect of Intervention

Shapiro-Wilk test of normality has shown that a *p* value was less than 0.05 for craniocervical flexion and all 8 subcategories of SF-36. As data were not normally distributed hence nonparametric tests were used for the within and between-group comparison.

Data for all outcomes at baseline, at second and fourth week, of the experimental group are presented in Table 1 and for the control group in Table 2.

There was a statistically significant difference between pre, mid, and posttreatment craniocervical flexion test scores in the experimental group. *Χ*2(2) = 78.28, *p* = 0.00.

Post hoc analysis with Wilcoxon signed-rank was conducted with Bonferroni correction applied, resulting in a significant level set at *p* < 0.017. Median (IQR) for pretreatment in the experimental group craniocervical flexion score was 21 (20 to 24), midtreatment was 24 (24 to 26), and posttreatment was 26 (24 to 28). There was a significant difference between pretreatment and midtreatment (*Z* = −5.56, *p* = 0.00), midtreatment and posttreatment (*Z* = −5.15, *p* = 0.00), and pretreatment and posttreatment (*Z* = −5.78, *p* = 0.00), showing that the craniocervical flexion score significantly improved after 2 weeks and further improved after 4 weeks of treatment in the experimental group.

There was a statistically significant difference between pre, mid, and posttreatment scores within all domains of SF 36 as *p* value < 0.05 when compared with the Friedman test. For post hoc analysis, Wilcoxon signed-rank was conducted with Bonferroni correction applied, resulting in a significant level set at *p* < 0.017 (for all 8 domains of SF 36) and there was significant difference between premid, midpost, and prepost treatment with *p* < 0.017 for all domain of SF-36 as shown in Table 1.

There was a statistically significant difference between pre, mid, and posttreatment craniocervical flexion test score in the control group *Χ*2 (2) = 68.70, *p* = 0.00.

Post hoc analysis with Wilcoxon signed-rank was conducted with Bonferroni correction applied, resulting in a significant level set at *p* < 0.017. Median (IQR) for pretreatment craniocervical flexion in the control group was 22 (20 to 24), midtreatment was 23 (22 to 26), and posttreatment was 24 (24 to 26). There was a significant difference between pretreatment and midtreatment (*Z* = −5.26, *p* = 0.00), midtreatment and posttreatment (*Z* = −4.66, *p* = 0.00), and pretreatment and posttreatment (*Z* = −5.53, *p* = 0.00), showing that craniocervical flexion was significantly improved after 2 weeks and further improved after 4 weeks of treatment in the control group.

There was a statistically significant difference between pre, mid, and posttreatment scores within all domains of SF 36 as *p* value < 0.05 when compared with the Friedman test. For post hoc analysis Wilcoxon signed-rank was conducted with Bonferroni correction applied, resulting in a significant level set at *p* < 0.017 (for all 8 domains of SF 36) and there was a significant difference between premid, midpost, and prepost treatment with *p* < 0.017 for all domain of SF-36 as shown in table 2.

Comparison of interquartile ranges and mean ranks of craniocervical flexion test score and eight domain of SF 36 between group 1 and group 2 has shown that there was no statistically or clinically significant difference in all eight domains of SF 36 at baseline, as value *p* > 0.05 and Cohen's *d* ≤ 0.25 for all variables as shown in Table 3.

There was a significant difference between both groups after the 2nd and 4th week as the mean rank for craniocervical flexion test score after the 2^nd^ week in the experimental group was 50.28 and in the control group was 38.72, while mean rank after 4 weeks in the experimental group was 51.60 and in the control group was 37.40 with value *p* < 0.05 and *d* ≥ 0.45, showing that neural mobilization is more effective in improving cervical muscle endurance than the conventional treatment as shown in Tables 4 and 5.

Comparison of both groups with Mann–Whitney *U* after two weeks of treatment has shown that there was a statistically significant difference between both groups in most of the domains of SF36 except physical functioning, role limitation due to emotional problems, and pain domain score. Mean rank for physical functioning domain after 2 weeks in the experimental group was 46.60 and in the control group was 42.40, mean rank for role limitation due to emotional problems after 2 weeks in the experimental group was 46.14 and in the control group was 42.86, while mean rank for pain domain after 2 weeks in the experimental group was 46.78 and in the control group was 42.22 with value *p* ≥ 0.05 and *d* ≤ 0.25 for these three domains are as shown in Table 4.

After the 4^th^ week, there was statistically and clinically significant improvement in almost all domains except in the pain domain of SF 36, in which there was no statistically significant difference but clinically significant difference was found as mean rank for the pain domain after 4 weeks in the experimental group was 49.43 and in the control group was 39.57 with value *p* = 0.065 and *d* = 0.39, while for all the other 7 domains of SF36 value *p* < .05, showing that neural mobilization is more effective in improving quality of life in patients of cervical radiculopathy as shown in Table 5.

## 4. Discussion

Debilitated persons with cervical radiculopathy are unable to perform their social obligations and show improper emotional behavior. Inability to do their physical tasks appropriately and loss of working hours affect the quality of life [2]. Among many treatment options discussed for cervical radiculopathy in the literature, conservative management is shown to be very effective as compared to surgical and pharmaceutical approaches. With advancement in health care, more attention has been given to conservative or nondrug treatment of cervical radiculopathy. Studies show that a multimodal approach may be more beneficial in alleviating these symptoms [5, 19].

Cervical radiculopathy often leads to inactivity, further deconditioning cervical muscles. Physical activity in the form of exercises is supported by evidence to enhance the physical, emotional, and cognitive functioning of an individual. This in turn impacts the quality of life, increases independence and reduces disability [13, 20]. Findings of these studies in literature correlates with the present study as there is a significant difference in cervical muscle endurance between both groups after the 2^nd^ and 4^th^ week of treatment, the mean rank for craniocervical flexion test score after 2 weeks in the experimental group is 50.28 and in the control group is 38.72, while mean rank after 4 weeks in the experimental group is 51.60 and in the control group is 37.40 with value *p* < 0.05 and *d* > 0.45. This shows that neural mobilization along with cervical isometrics is more effective in improving cervical muscle endurance than the conventional treatment. Hypoalgesic effect of isometric exercises is also found in study conducted by Ojoawo and Olabode [21].

In literature, it is evident that neural mobilization can be used as a standalone approach or along with other exercises. When combined treatment is provided it shows promising results. The study by Savva et al. has demonstrated improvement in grip strength, pain, disability, and cervical range of motion when people with cervical radiculopathy were treated with neural mobilization and cervical traction [22].

Additionally, neurophysiological and analgesic effect of neural mobilization predicts pain relief and improves cervical functioning. It works by stimulating mechanical receptors, reducing edema, and improving circulation. A study done by Lima and Abner suggests that exercise is an integral part of rehabilitation of patients suffering from musculoskeletal disorders as it promotes exercise induced analgesia. Cleland et al. predicted short term successful outcomes in cervical radiculopathy by applying manual therapy, cervical traction, and deep neck flexor muscle strengthening exercises [23–25]. Conclusion of the mentioned studies are in consistent with present study as within-group comparison has shown that there is statistically significant difference between pre, mid, and posttreatment scores within all domain of SF 36 in both groups, showing that both interventions are effective in improving quality of life in subjects with cervical radiculopathy, while between-group comparison has shown that all variables were similar at baseline but after 4 weeks of treatment there was statistically and clinically significant improvement in almost all domains of SF 36 in the experimental group. Improvement in physical and emotional components is indication of improvements in quality of life, showing that neural mobilization is more effective in improving quality of life in patients of cervical radiculopathy. Neurodynamic intervention has also shown to improve neuropathic symptoms by exerting their therapeutic effects [26].

In previous studies, little attention is paid on measuring the quality of life of a patient with cervical radiculopathy. This study analyzes the effects of exercises and neural mobilization on the quality of life of patients by considering all physical and mental components. Results of this study also depict that multimodal management which comprises of neurodynamic mobilization and exercises is more effective as compared to conservative treatment in cervical radiculopathy.

### 4.1. Limitations

In combined treatment it is difficult to interpret the results of a single intervention, and while inferring strength-related results, physical components of both genders should be considered. This may be considered as the limitations of this study. The sample was collected from a single setting so results cannot be generalized. Also, objective measurements like dysesthesia, weakness of upper extremity muscles, and radiating pain were not collected. However, further research is required to determine if it is clinically worthwhile and what will be the effect of modification in the regime.

## 5. Conclusion

Neural mobilization combined with cervical exercises shows more significant effects in improving quality of life and endurance in patients with cervical radiculopathy than cervical isometric exercises alone.

## Figures and Tables

**Figure 1:** The figure for a parallel design.

**Table 1:** Comparison of craniocervical flexion test and 8 domains of SF 36 within the experimental group.

Variable	—	Interquartile range	Mean rank^a^	Chi-square (*X*^2^), *p* value^a^	Post hoc analysis	*Z* score^b^	*p* value^b^
Craniocervical flexion (mmHg)	Base line	21 (20 to 24)	1.07	78.28, *p* < 0.05	Pre and midtreatment	-5.56	<0.017
	After 2^nd^ week	24 (24 to 26)	2.10		Mid and posttreatment	-5.15	<0.017
	After 4^th^ week	26 (24 to 28)	2.83		Pre and posttreatment	-5.78	<0.017
Physical functioning–SF36	Baseline	35 (20 to 55)	1.15	73.92, *p* < 0.05	Pre and midtreatment	-4.59	<0.017
	After 2^nd^ week	57 (35 to 70)	1.94		Mid and posttreatment	-5.43	<0.017
	After 4^th^ week	75 (60 to 85)	2.91		Pre and posttreatment	-5.46	<0.017
Role limitation due to physical health–SF36	Baseline	0 (0 to 25)	1.28	66.72. *p* < 0.05	Pre and midtreatment	-4.38	<0.017
	After 2^nd^ week	25 (25 to 50)	1.91		Mid and posttreatment	-5.01	<0.017
	After 4^th^ week	62.5 (50 to 100)	2.81		Pre and posttreatment	-5.49	<0.017
Role limitation due to emotional problem–SF36	Baseline	0 (0 to 33.3)	1.59	36.20, *p* < 0.05	Pre and midtreatment	-2.68	<0.017
	After 2^nd^ week	33.3 (0 to 66.7)	1.89		Mid and posttreatment	-3.72	<0.017
	After 4^th^ week	66.7 (33.3 to 100)	2.52		Pre and posttreatment	-4.49	<0.017
Energy/fatigue–SF36	Baseline	45 (35 to 50)	1.18	61.82, *p* < 0.05	Pre and midtreatment	-4.56	<0.017
	After 2^nd^ week	55 (45 to 60)	2.03		Mid and posttreatment	-4.95	<0.017
	After 4^th^ week	60 (50 to 75)	2.78		Pre and posttreatment	-5.21	<0.017
Emotional wellbeing–SF36	Baseline	52 (44 to 60)	1.45	36.96, *p* < 0.05	Pre and midtreatment	-3.83	<0.017
	After 2^nd^ week	56 (52 to 64)	1.94		Mid and posttreatment	-4.30	<0.017
	After 4th week	66 (53 to 75)	2.60		Pre and posttreatment	-4.61	<0.017
Social functioning–SF36	Baseline	43.75 (37.5 to 62.5)	1.38	53.26, *p* < 0.05	Pre and midtreatment	-3.91	<0.017
	After 2^nd^ week	62.50 (50 to 75)	1.89		Mid and posttreatment	-5.06	<0.017
	After 4^th^ week	75 (62.5 to 87.5)	2.74		Pre and posttreatment	-4.95	<0.017
Pain–SF36	Baseline	45 (43.1 to 45)	1.34	61.10, *p* < 0.05	Pre and midtreatment	-4.26	<0.017
	After 2^nd^ week	55 (45 to 66.87)	1.92		Mid and posttreatment	-4.97	<0.017
	After 4^th^ week	67.5 (55 to 86.87)	2.74		Pre and posttreatment	-5.17	<0.017
General health–SF36	Baseline	40 (35 to 55)	1.34	63.18, *p* < 0.05	Pre and midtreatment	-3.79	<0.017
	After 2^nd^ week	52.5 (40 to 65)	1.76		Mid and posttreatment	-5.54	<0.017
	After 4^th^ week	75 (50 to 83.75)	2.90		Pre and posttreatment	-5.56	<0.017

^a^ Friedman test statistics, ^b^ post hoc analysis.

**Table 2:** Comparison of craniocervical flexion test and 8 domains of SF 36 within the control group.

Variable	—	Interquartile range	Mean rank^a^	Chi-square (*X*^2^), *p* value^a^	Post hoc analysis	*Z* score^b^	*p* value^b^
Craniocervical flexion (mmHg)	Base line	22 (20 to 24)	1.18	68.70, *p* < 0.05	Pre and midtreatment	-5.26	<0.017
	After 2^nd^ week	23 (22 to 26)	2.09		Mid and posttreatment	-4.66	<0.017
	After 4^th^ week	24 (24 to 26)	2.73		Pre and posttreatment	-5.53	<0.017
Physical functioning–SF36	Baseline	40 (21.25 to 55)	1.41	54.25, *p* < 0.05	Pre and midtreatment	-3.17	0.001
	After 2^nd^ week	52.5 (30 to 65)	1.86		Mid and posttreatment	-5.03	<0.017
	After 4^th^ week	70 (45 to 80)	2.73		Pre and posttreatment	-4.66	<0.017
Role limitation due to physical health–SF36	Baseline	0 (0 to 0)	1.63	37.90, *p* < 0.05	Pre and midtreatment	-2.55	0.011
	After 2^nd^ week	0 (0 to 25)	1.88		Mid and posttreatment	-4.11	<0.017
	After 4^th^ week	50 (0 to 75)	2.50		Pre and posttreatment	-4.45	<0.017
Role limitation due to emotional problem–SF36	Baseline	16.65 (0 to 66.70)	1.88	17.03, *p* < 0.05	Pre and midtreatment	-1.41	0.157
	After 2^nd^ week	16.65 (0 to 66.70)	1.92		Mid and posttreatment	-2.75	<0.017
	After 4^th^ week	66.70 (0 to 100)	2.20		Pre and posttreatment	-2.88	<0.017
Energy/fatigue–SF36	Baseline	42.5 (35 to 50)	1.42	48.42, *p* < 0.05	Pre and midtreatment	-4.01	<0.017
	After 2^nd^ week	45 (36.25 to 55)	1.94		Mid and posttreatment	-4.47	<0.017
	After 4^th^ week	55 (45 to 63.75)	2.64		Pre and posttreatment	-4.93	<0.017
Emotional wellbeing–SF36	Baseline	52 (40 to 56)	1.61	27.22, *p* < 0.05	Pre and midtreatment	-2.64	<0.017
	After 2^nd^ week	52 (40 to 60)	1.92		Mid and posttreatment	-4.04	<0.017
	After 4^th^ week	60 (48 to 60)	2.47		Pre and posttreatment	-4.13	<0.017
Social functioning–SF36	Baseline	50 (37.5 to 62.5)	1.63	35.89, *p* < 0.05	Pre and midtreatment	-2.44	0.015
	After 2^nd^ week	50 (37.5 to 62.5)	1.85		Mid and posttreatment	-4.37	<0.017
	After 4^th^ week	62.5 (50 to 75)	2.52		Pre and posttreatment	-4.45	<0.017
Pain–SF36	Baseline	45 (45 to 45)	1.45	54.60, *p* < 0.05	Pre and midtreatment	-3.37	<0.017
	After 2^nd^ week	45 (45 to 67.5)	1.83		Mid and posttreatment	-4.45	<0.017
	After 4^th^ week	55 (55 to 77.5)	2.72		Pre and posttreatment	-5.13	<0.017
General health perception–SF36	Base line	35 (31.25 to 45)	1.41	51.95, *p* < 0.05	Pre and midtreatment	-3.64	<0.017
	After 2^nd^ week	40 (35 to 50)	1.92		Mid and posttreatment	-4.58	<0.017
	After 4^th^ week	47.5 (40 to 60)	2.67		Pre and posttreatment	-5.01	<0.017

**Table 3:** Comparison of the baseline craniocervical flexion and 8 domain of SF 36 between the experimental and control group.

Variable	Group (*n* = 88) Experimental = 44 Control = 44	Baseline IQR	Baseline mean ranks	Man Whitney U	Sig. (2-tailed) and effect size (Cohen's *D*)
Craniocervical flexion	Experimental	21 (20 to 24)	42.24	868.50	*p* = 0.381, *d* = 0.178
	Control	22 (20 to 24)	46.76		
Physical functioning–SF36	Experimental	35 (20 to 55)	42.82	894.0	*p* = 0.534, *d* = 0.132
	Control	40 (21.25 to 55)	46.18		
Role limitation due to physical health–SF36	Experimental	0 (0 to 25)	46.30	889.0	*p* = 0.395, *d* = 0.141
	Control	0 (0 to 0)	42.70		
Role limitation due to emotional problem–SF36	Experimental	0 (0 to 33)	42.73	890.0	*p* = 0.480, *d* = 0.139
	Control	16.65 (0 to 66.7)	46.27		
Energy/fatigue–SF36	Experimental	45 (30.5 to 50)	44.69	959.50	*p* = 0.943, *d* = 0.016
	Control	42.5 (35 to 50)	44.31		
Emotional wellbeing–SF36	Experimental	52 (44 to 60)	46.73	870.0	*p* = 0.410, *d* = 0.175
	Control	52 (40 to 56)	42.27		
Social functioning–SF36	Experimental	43.75 (37.5 to 62.5)	42.94	899.50	*p* = 0.556, *d* = 0.122
	Control	50 (37.5 to 62.5)	46.6		
Pain–SF36	Experimental	45 (43.12 to 45)	43.24	912.50	*p* = 0.612, *d* = 0.099
	Control	45 (45 to 45)	45.76		
General health perception–SF36	Experimental	40 (35 to 55)	47.76	824.50	*p* = 0.223, *d* = 0.25
	Control	35 (31.25 to 45)	41.24		

**Table 4:** Comparison of the craniocervical flexion and 8 domain of SF 36 between the experimental and control group after 2 weeks of treatment.

Variable	Group (*n* = 88) Experimental = 44 Control = 44	After 2^nd^ week IQR	After 2^nd^ week mean ranks	Man Whitney *U*	Sig. (2-tailed)
Craniocervical flexion	Experimental	24 (24 to 26)	50.28	713.5	*p* = 0.029, *d* = 0.465
	Control	23 (22 to 26)	38.72		
Physical functioning–SF36	Experimental	57.5 (35 to 70)	46.6	875.50	*p* = 0.439, *d* = 0.165
	Control	52.5 (30 to 65)	42.4		
Role limitation due to physical health–SF36	Experimental	25 (25 to 50)	53.3	581.0	*p* = 0.01, *d* = 0.733
	Control	0 (0 to 25)	35.7		
Role limitation due to emotional problem–SF36	Experimental	33.3 (0 to 66.7)	46.14	896.00	*p* = 0.526, *d* = 0.128
	Control	16.65 (0 to 66.7)	42.86		
Energy/fatigue–SF36	Experimental	55 (45 to 60)	50.6	699.50	*p* = 0.023, *d* = 0.493
	Control	45 (36.25 to 55)	38.4		
Emotional wellbeing–SF36	Experimental	56 (52 to 64)	52.47	617.50	*p* = 0.003, *d* = 0.657
	Control	52 (40 to 60)	36.53		
Social functioning–SF36	Experimental	62.5 (50 to 75)	50.03	724.50	*p* = 0.037, *d* = 0.445
	Control	50 (37.5 to 62.5)	38.97		
Pain–SF36	Experimental	55 (45 to 68.87)	46.78	867.50	*p* = 0.382, *d* = 0.18
	Control	45 (45 to 67.5)	42.22		
General health perception–SF36	Experimental	52.5 (40 to 65)	52.99	594.50	*p* = 0.002, *d* = 0.706
	Control	40 (35 to 50)	36.01		

**Table 5:** Comparison of the craniocervical flexion and 8 domain of SF 36 between the experimental and control group after 4 weeks of treatment.

Variable	Group (*n* = 88) Experimental = 44 Control = 44	After the 4^th^ week IQR	After 4^th^ week mean ranks	Man Whitney *U*	Sig. (2-tailed)
Craniocervical flexion	Experimental	26 (24 to 28)	51.6	655.5	*p* = 0.007, *d* = 0.579
	Control	24 (24 to 26)	37.4		
Physical functioning–SF36	Experimental	75 (60 to 85)	51.3	669.0	*p* = 0.012, *d* = 0.552
	Control	70 (45 to 80)	37.70		
Role limitation due to physical health–SF36	Experimental	62.5 (50 to 100)	51.99	638.50	*p* = 0.05, *d* = 0.613
	Control	50 (0 to 75)	37.01		
Role limitation due to emotional problem–SF36	Experimental	66.7 (33.3 to 100)	50.02	725.0	*p* = 0.035, *d* = 0.443
	Control	66.7 (0 to 100)	38.98		
Energy/fatigue–SF36	Experimental	60 (50 to 75)	51	682.0	*p* = 0.016, *d* = 0.526
	Control	55 (45 to 63.75)	38		
Emotional wellbeing–SF36	Experimental	66 (53 to 75)	52.48	617.0	*p* = 0.003, *d* = 0.657
	Control	60 (48 to 60)	36.52		
Social functioning–SF36	Experimental	75 (62.5 to 87.5)	53.14	588.00	*p* = 0.001, *d* = 0.718
	Control	62.5 (50 to 75)	35.86		
Pain–SF36	Experimental	67.5 (55 to 86.87)	49.43	751.00	*p* = 0.065, *d* = 0.393
	Control	55 (55 to 77.5)	39.57		
General health perception–SF36	Experimental	75 (50 to 83.75)	55.59	480.00	*p* = 0.00, *d* = 0.964
	Control	47.5 (40 to 60)	33.41		

## Data Availability

Data will be available on request.

## Additional Points

*Key Messages*. (i) What is already known on this topic? The quality of life of persons with cervical radiculopathy is affected because of the limitations in their social, emotional, and work life. In literature, there are many treatment options available for cervical radiculopathy including neural mobilization which has shown promising results. But little attention is paid towards measuring the quality of life of these persons. (ii) What does this study add? As the cost-effective treatment option techniques mentioned in this study can help people with cervical radiculopathy, there is a nonavailability of expensive modalities. This can also be utilized to change the treatment protocols in clinical practice.
